The article "Reinforcement Learning in Neurocritical and Neurosurgical Care: Principles and Possible Applications" was published in 2021. Journal: Comput Math Methods Med.

# Reinforcement Learning in Neurocritical and Neurosurgical Care: Principles and Possible Applications

**DOI:** 10.1155/2021/6657119

**Published:** 2021-02-22

**Authors:** Ying Liu, Nidan Qiao, Yuksel Altinel

**Affiliations:** ^1^Lhorong People's Hospital, Tibet, China; ^2^Department of Neurosurgery, Huashan Hospital, Shanghai Medical School, Fudan University, Shanghai, China; ^3^Shanghai Clinical Medical Center of Neurosurgery, Shanghai, China; ^4^Neurosurgical Institute of Fudan University, Shanghai, China; ^5^Medical Science in Clinical Investigation, Harvard Medical School, Boston, USA

## Abstract

Dynamic decision-making was essential in the clinical care of surgical patients. Reinforcement learning (RL) algorithm is a computational method to find sequential optimal decisions among multiple suboptimal options. This review is aimed at introducing RL's basic concepts, including three basic components: the state, the action, and the reward. Most medical studies using reinforcement learning methods were trained on a fixed observational dataset. This paper also reviews the literature of existing practical applications using reinforcement learning methods, which can be further categorized as a statistical RL study and a computational RL study. The review proposes several potential aspects where reinforcement learning can be applied in neurocritical and neurosurgical care. These include sequential treatment strategies of intracranial tumors and traumatic brain injury and intraoperative endoscope motion control. Several limitations of reinforcement learning are representations of basic components, the positivity violation, and validation methods.

## 1. Introduction

Dynamic decision-making was essential in the clinical care of surgical patients. It is often difficult to determine treatment dosage precisely or decide whether to start or stop treatment in specific situations (e.g., fluid therapy in patients with electrolytes disturbance or anticoagulation after surgery). Doctors often made multiple sequential decisions according to their medical experience. The unmet clinical need falls into whether we can develop a sequential clinical decision-making support system (dynamic treatment regime (DTR)) to better aid doctors such that it can improve patients' outcomes. A DTR comprises a sequence of decision rules, one per stage of intervention, that recommends how to individualize treatment to patients based on evolving treatment and covariate history. For example, in the case of a patient with traumatic brain injury (TBI) and intracranial hypertension (Figure 1(a)), should we apply concentrated sodium? Should the patient be put on mechanical ventilation later? Should the patient be sedated to alleviate airway resistance? How can we treat patients so that their outcomes are as good as possible?

The majority of comparative effectiveness studies compared two treatment modalities on a single timepoint to find better treatment and potential treatment modifications. For sequential treatments in multiple stages (Figure 1(b)), recent advances in statistical and computational science provided the opportunity to identify the optimal strategy.

The reinforcement learning (RL) algorithm finds sequential optimal decisions among multiple suboptimal options, which can solve the above problem [1]. Reinforcement learning was considered a third type of machine learning algorithm besides supervised learning and unsupervised learning, which has its own set of challenges and methods. To integrate reinforcement learning into healthcare, it is essential first to understand how the algorithm works. This review is aimed at introducing the basic idea as well as the pros and cons of reinforcement learning. We also reviewed the literature of existing practical applications of reinforcement learning and proposed several potential aspects where it can be applied in neurocritical and neurosurgical care.

## 2. Principles of RL

In computer science, RL's classic problem is to apply horizontal forces (to the left or the right) on a cart that can move left or right on a track to keep a pole hinged to the car from falling off the initial vertical position. The computer starts to experiment by giving the cart a force. If the pole was kept hinged, the computer gets the reward (e.g., plus one). If a failure occurs, then the computer has to restart a new episode. By doing this experiment repeatedly, the computer learns how to achieve the goal finally [2]. The whole process is the RL algorithm.

Several uniform conceptions are introduced in this scenario: the state, the action, and the reward (Figure 2). The state (S) is the status a patient is at a specific time point, including vital signs, lab tests, physical examinations, intracranial pressure, demographics, and the dosage of medications. The action (A) is the treatment physicians give, or the patient receives at that time point, e.g., concentrated sodium or mechanical ventilation. The reward (R) is the response that the patient reacts to the action. Strategy is the combination of sequential actions through time, e.g., how a physician would treat a patient in the whole in-hospital duration. Environment is the external system with which the patient interacts (that is the medical knowledge we have).

Then, we define the DTR as the treatment prediction function that takes the current state and translates it into action. The ultimate goal of reinforcement learning was to find the optimal DTR (best treatment combination throughout a patient's trajectory) that maximizes the expected total reward from all actions performed (e.g., keep the intracranial pressure in the normal range, Figure 1(b)).

In the previous computer example, the computer can repeatedly play the game and update the algorithm parameters based on real-time outcomes [2]. In most medical practices, we cannot wait until we observe the previous patient's efficacy to decide the next patient's treatments, except we are doing an adaptive trial. Most of the reinforcement learning studies in the medical area are called batch reinforcement learning or offline reinforcement learning, in which a fixed dataset is all that is available, and a real-time environment is not accessible.

## 3. Studies Using RL Algorithms

Reinforcement learning studies can be further categorized as a statistical RL study and a computational RL study. The reasons for using statistical RL and computational RL to classify literature are that these two subgroups use different estimation methods and are applied in different kinds of dataset.

### 3.1. Statistical RL

A statistical RL study extends a usual one-stage two-treatment comparison into two stages, which was first studied and implemented to reanalysis sequential multiple assignment randomized trials (SMART) [3]. SMART involves initial randomization of patients to possible treatment options, followed by rerandomizing the patients at each subsequent stage to other treatment options available at that stage. Examples of studies using SMART design (or its precursors) include the Clinical Antipsychotic Trials of Intervention Effectiveness (CATIE) for Alzheimer's disease [4], the Sequenced Treatment Alternatives to Relieve Depression (STARD) trial [5], a 2-stage trial designed to reduce mood and neurovegetative symptoms among patients with malignant melanoma [6], several trials that evaluated immune checkpoint inhibitors [7], and dynamic monitoring strategies based on CD4 cell counts [8]. In nonrandomized observational studies, Moodie et al. extended this method to observational data in a breastfeeding research to investigate any breastfeeding habits' effect on verbal cognitive ability [9]. Chen et al. also used the RL method in observation data to find the optimal dosage in warfarin treatment. They found that the dose should be increased if patients were taking cytochrome P450 enzyme inhibitors [10]. Statistical RL studies were usually solved by fitting linear outcome models in a recursive manner. More recently, some other methods have been developed such as inverse probability weighted estimator and augmented inverse probability weighted estimator [11, 12].

### 3.2. Computational RL

Computational RL deals with problems in the realm with higher dimensions, which means multiple treatment options within multiple stages [13, 14]. Martín-Guerrero et al. used RL to learn a policy for erythropoietin prescription to maintain patients within a targeted hemoglobin range and proposed a methodology based on RL to optimize erythropoietin therapy in hemodialysis patients [15, 16]. Parbhoo et al. proposed an RL algorithm to assign the most appropriate treatment to HIV patients. They found that the proposed algorithm had the highest accumulated long-term rewards over five years [17]. Liu et al. proposed a deep reinforcement learning framework to prevent graft versus host disease [18]. The most recent published RL study was by Komorowski et al., and they predicted optimal fluid therapy and vasopressor usage in sepsis patients, which was validated in an independent database [19]. Other studies also suggested that computational RL can be used in treatment optimization. Nemati et al. presented a clinical sequential decision-making framework to adjust individualized warfarin dosing for stabilizing thromboplastin time [20]. Ribba et al. recommended a personalized regime of medication dosage [21]. Zhu et al. developed a double Q-learning with a dilated recurrent neural network for closed-loop glucose control in type 1 diabetes mellitus [22]. Recently, Ge et al. integrated reinforcement learning and recurrent neural network to explore public health intervention strategies [23]. Computational RL requires large amount of data during dynamic programming and thus is not suited for randomized trials with limited sample. [24, 25]

## 4. Proposed Aspects of Neurosurgical and Neurocritical Care

Effective chemotherapy dosing policies and automated radiation adaptation protocols after surgical resection of the intracranial malignant tumor could be solved using reinforcement learning. Similarly, in patients with benign tumors, e.g., growth hormone secreting pituitary adenomas, the optimal treatment sequences, including medication, radiation, and surgery, were unknown.

The method proposed by Brett et al. that RL could manage optimal control of propofol-induced hypnosis during anesthesia practice [13] could potentially be applied during the anesthesia process in neurosurgeries. Moreover, researchers were developing surgical robots using reinforcement learning, including creating a colon endoscope robot that could adjust its locomotion [26] and a gesture recognition algorithm for hand-assisted laparoscopic surgery [27]. All these studies suggested that reinforcement learning was an efficient approach to solving control problems by interacting with the environment and acquiring the optimal control policy. A similar idea could be applied to neuroendscope during transventricular surgeries and transnasal surgeries.

Regarding the whole treatment process of a patient, two recent papers also proposed using RL to design clinical supporting tools for plastic surgery and gastric intestinal surgeries [26, 28]. Similarly, in neurocritical care, reinforcement learning can also be applied to determine optimal postsurgical management, e.g., precise fluid volumes were essential for electrolyte management in patients with electrolyte disturbance after surgery. Moreover, TBI's entire treatment trajectory could be modeled by a reinforcement learning framework, as depicted in Figure 3. An algorithm interacts with its environment (data from electronic health records) to represent states (disease acuity), actions (treatment), and the ultimate goal (such as survival). This algorithm applies to a patient presenting with TBI and estimates the clinical utility of observation, intracranial pressure monitoring, or craniotomy. The process identifies the best treatments at each stage that are most likely to achieve the ultimate goal.

## 5. Limitations of Reinforcement Learning

Though reinforcement learning was promised to solve dynamic treatment problems, several limitations hindered extensive applying this special algorithm in clinical research.

The first step in applying reinforcement learning to a healthcare problem is to collect and preprocess accurate medical data. Most existing work defines the states with raw physiological, pathological, and demographic information. We should bear in mind that unmeasured or unobserved states might also affect clinical decisions, e.g., the surgeons' preference. Moreover, how to categorize treatment with continuous presentations, e.g., infusion volume, needs further discussion. The reward may be at the core of a reinforcement learning process. Sometimes, it was easy to define the reward both in the intermediate state and the final state, e.g., INR in warfarin adjustment or blood glucose in optimal diabetes mellitus control. While in most medical settings, the outcomes of treatments cannot be naturally generated and explicitly represented, e.g., the reward was defined as a function of viral load, CD4+ count, and the number of mutations in an HIV study [17]. The reward was defined by a complex function of vital signs and intubation status in an intubation weaning study [20].

Like any other casual inference studies, the violation of positivity (the conditional probability of receiving each treatment is greater than zero) is a major limitation in training the reinforcement learning algorithm. For example, in patients with severe hyponatremia, treatment options include “no action,” “normal saline,” and “3% concentrated sodium,” and physicians always treat these patients with concentrated sodium. Generally, we know that we cannot do the “no action” or the “normal saline” option because it makes no sense. However, some patients still had no improvement on serum sodium despite optimal medical management by human clinicians. Since the reinforcement learning algorithm can learn to avoid dosing patients or acting differently than the clinician in severe cases to avoid being punished, the reinforcement learning algorithm might choose the “no action” or the “normal saline” option in such cases. Omer et al. also mentioned in their guideline that reinforcement learning algorithms' quality depends on the number of patient histories for which the proposed and actual treatment policies agree [29].

It is essential to estimate how the learned policies might perform on retrospective data before testing them in real clinical environments. Current validations in reinforcement learning literature were based on either the internal dataset (where the algorithm was obtained) or the external dataset (an independent dataset) [19]. The basic idea behind validation was to compare the total reward generated by the reinforcement learning algorithm and the total reward from the actual treatment. Unlike other board/video games, in a clinical setting, physicians cannot and are not allowed to play out a large number of scenarios to learn the optimal policy. Further validation of the algorithm needs randomizing patients treated under the algorithm's policy versus treated under the clinician's policy.

## 6. Conclusion

In conclusion, reinforcement learning algorithm is an emerging method to find an optimal treatment regime during clinical decision-making. Proposed neurosurgical and neurocritical applications include sequential treatment of intracranial tumors and traumatic brain injury. Future aspects also involve intraoperative motion control. Limitations of reinforcement learning warrant further collaborations of both computational scientists and physicians.

## Figures and Tables

**Figure 1:** (a) A patient with traumatic brain injury and intracranial hypertension; sequential treatment includes concentrated sodium, mechanical ventilation, sedation, and possible outcomes. (b) The trajectories (strategies) of three patients and their expected total reward from all treatments performed.

**Figure 2:** Uniform conceptions in reinforcement learning: the state, the action, and the reward. Physicians gave treatment (action, A) to the patient (state, S) with some vital signs, lab tests, and physical examinations at a specific time point. The patient responds to the treatment (reward, R).

**Figure 3:** Illustration of a proposed reinforcement learning framework to find optimal dynamic treatment therapy in patients with traumatic brain injury. *P* represents the probability of the outcome after treatment at each stage; *r* represents the reward after treatment at each stage.
